The article "Efficacy and Safety of Bifidobacterium Quadruple Viable Bacteria Combined with Mesalamine against UC Management: A Systematic Review and Meta-Analysis" was retracted in 2023. Reasons: signs of a paper mill; compromised peer review; unreliable results or conclusions.

# Efficacy and Safety of Bifidobacterium Quadruple Viable Bacteria Combined with Mesalamine against UC Management: A Systematic Review and Meta-Analysis

**DOI:** 10.1155/2022/8272371

**Published:** 2022-10-04

**Authors:** Fei Xie, Shichao Li, Yao Fan, Wusheng Li, Qijun Lv, Xin Sun, Yingshuang Chen, Xiangdong Yang

**Affiliations:** ^1^The Affiliated Traditional Chinese Medicine Hospital of Southwest Medical University, China; ^2^Southwest Medical University, China; ^3^The Affiliated Traditional Chinese Medicine Hospital of Southwest Medical University, Chengdu Anorectal Hospital, Colorectal and Anal Surgery, China

## Abstract

**Objective:**

To systematically assess effectiveness and safety of Bifidobacterium quadruple viable bacteria combined with mesalamine against ulcerative colitis (UC) in the Asian population.

**Methods:**

An electronic search was conducted in PubMed, Embase, Cochrane Library, CNKI, VIP, and Wanfang databases for a random collection of controlled trials of Bifidobacterium quadruple viable bacteria combined with mesalamine against UC. Following data screening and extraction, a Cochrane risk assessment tool was adopted to evaluate the quality of the included studies, and RevMan 5.3 and Stata/SE 15.1 software were used for meta-analysis.

**Results:**

Nineteen articles which enrolled 1,707 subjects were included ultimately in this study. The experimental group performed better than the control group in improving the Mayo score (MD = −1.94, 95% CI = (−2.69, −1.19), *P* < 0.00001), increasing the total clinical efficiency (OR = 5.10, 95% CI (3.53, 7.38), *P* < 0.00001), reducing the levels of IL-8 (SMD = −1.79, 95% CI (-2.36, -1.12), *P* < 0.00001), increasing the levels of IL-4 (SMD = 1.00, 95% CI (0.60, 1.41), *P* < 0.00001), and reducing the levels of hsCRP (MD = −3.26, 95% CI (-4.28, -2.25), *P* < 0.00001), TNF-*α* (MD = −7.11, 95% CI (-9.23, -5.00), *P* < 0.00001), ox-LDL (MD = −14.46, 95% CI (-17.20, -11.72), *P* < 0.00001), and LPO (MD = −3.55, 95% CI (-4.70, -2.39), *P* < 0.0001) as well as increasing SOD level (SMD = 1.68, 95% CI (1.02, 2.35), *P* < 0.00001), and adverse reactions were substantially less than that of control (OR = 0.43, 95% CI = (0.28, 0.66), *P* = 0.0001).

**Conclusion:**

In conclusion, the current meta-analysis shows that Bifidobacterium quadruple viable bacterium combined with mesalamine has a satisfactory effect in the treatment of UC in China, and its safety is better than that of mesalamine or Bifidobacterium quadruple viable bacteria alone. However, randomized controlled trials with standardized designs and large sample sizes are still needed for further validation.

## 1. Introduction

Ulcerative colitis (UC) represents a chronic nonspecific inflammation in the intestinal tracts with uncertain etiology, and it has a long course of disease, recurrent episodes, and difficult treatment [1]. UC lesions are mainly in the colon, and superficial mucosal inflammation begins from the rectum and extends proximally, usually leading to intestinal mucosal ulceration, hemorrhage, fulminant colitis, and toxic megacolon [2]. Factors related to the incidence of UC mainly include diet, drugs, lifestyle, genetic factors, and immune disorders, which may affect the intestinal microbes of patients or the immune response to antigens [3, 4]. In recent years, UC occurrence has shown a global increase with the development of the global economy [5]. Hospitalization due to UC in China has also shown an increasing trend in recent years [6], and the situation has gradually become more frequent with the prolongation of the disease course [7]. Therefore, it is necessary to explore effective treatments for UC.

Mesalamine is a 5-aminosalicylic acid drug, while 5-aminosalicylic acid is a first-line therapy for mild to moderate UC [8, 9]. A meta-analysis of oral, topical, or combined both medication with mesalamine illustrated that it is safe and well-tolerated in UC treatment in patients who responded well to mesalamine [10]. Despite mesalamine has achieved certain effects against UC, there are potential side effects and poor efficacy in some patients [11–13]. It is therefore that a combination of medications is needed for UC management.

Currently, increasing researchers highlight the role of intestinal flora for UC treatment. The intestinal flora has its diversity, and the balance of beneficial and pathogenic bacteria has a close association with pathogenesis, prognosis, and recurrence of UC. Studies have shown that the intestinal microbiota composition and the clinical course of UC are correlated, and for the recurrence rate of UC in the remission stage and the treatment in the active stage, the composition of intestinal microbiota and the decrease of the diversity of some microorganisms are also connected to a later clinical course of UC [14]. Several trials have found that improvement of UC can be achieved by intervention to improve intestinal flora [15–21]. Bifidobacterium quadruple viable bacterium, a type of quadruple live immunomodulator, has been tested and proved to have satisfactory effect and safety in combination with mesalamine in treating UC [22–30].

A growing number of clinical trials have been conducted to verify whether mesalamine in combination with Bifidobacterium quadruple viable bacteria can exert a desired efficacy and safety during UC treatment, whereas most trials are small samples, and the efficacy and safety are still controversial. Therefore, a systematic review and meta-analysis was conducted in the current research to address the safety and efficacy of mesalamine combined with Bifidobacterium quadruple viable bacteria in treating UC, expecting to offer some proofs for the management of UC in future.

## 2. Materials and Methods

The current work is a systematic review and meta-analysis, which is performed as per the Preferred Reporting Items for Systematic Reviews and Meta-Analysis guidelines. It has been registered to The International Prospective Register of Systematic Reviews (CRD42022337822).

### 2.1. Inclusion Criteria

(1) Research subjects: adult patients with UC. (2) Interventions: the control group was treated with mesalamine or Bifidobacterium quadruple viable bacteria alone; the experimental group received a combination of mesalamine and Bifidobacterium quadruple viable bacteria. (3) The primary results were Mayo score, response rate, and interleukins, and secondary results were TNF-*α*, hypersensitive c-reactive protein (hs-CRP), ox-LDL, LPO, SOD, and adverse reactions. (5) The study type was randomized controlled trial.

### 2.2. Exclusion Criteria

(1) Non-RCTs. (2) Use of other microecological agents in the intervention. (3) Too low quality or serious errors in design. (4) Duplicate published literature, conference abstracts, and reviews.

### 2.3. Literature Retrieval

Databases CNKI, PubMed, Cochrane Library, Embase, VIP, and Wanfang were used for retrieval of the relevant literature from the inception of each database to December 30, 2021. Subject terms applied for the search were input together with free words. Taking PubMed as an example, “Mesalamine”, “Bifidobacterium”, “Colitis”, and “Ulcerative” were adopted as subject terms.

### 2.4. Literature Screening and Data Extraction

The literature was screened and data were extracted by two independent researchers (XF and LSC) using EndNote X9 as per inclusion and exclusion criteria. Meanwhile, cross-validation was also performed. When discrepancies occurred, a third investigator assisted in reaching an agreement. The collected content included first author, publication date, trial sample size, mean age, intervention, duration of treatment, and outcome measures.

### 2.5. Literature Quality Evaluation

The literature quality was assessed independently by two researchers based on Cochrane risk of bias tools in Handbook 5.1.0 [31], and a third party was consulted in case of discrepancies. The assessment included the following: the method of random sequence generation and the technique of allocation concealment; the implementation of blinding in randomized trials such as investigators, subjects, and outcome assessors; the outcome data integrity; the presence or absence of selective reporting of results; and the presence or absence of other biases.

### 2.6. Statistical Analysis

A meta-analysis was carried out through RevMan 5.3 software. Counting data were expressed as relative risk ratio (RR), and measurement data were expressed as mean difference (MD) or standardized mean difference (SMD), with 95% confidence interval. *I*^2^ tests were employed to determine the presence of heterogeneity, with *I*^2^ less than or equal to 50% or *P* more than 0.05 indicating good homogeneity, and a fixed-effects model was subsequently adopted. When *I*^2^ or *P* value was not within the specific range, a random-effects model was adopted. The literature was ruled out one by one to perform sensitivity analysis. Subgroup analysis was performed when it was necessary to figure out the source of heterogeneity. Stata/SE 15.1 software was used to detect publication bias using Begger's and Egger's tests. The value of *P* > 0.05 was considered as insignificant publication bias, while *P* < 0.05 indicated publication bias was significant. If publication bias existed, the trim and filling method was supplemented.

## 3. Results

### 3.1. Literature Retrieval Process

The initial search yielded 336 articles, 109 in Chinese and 227 in English, and 19 articles were finally included through screening, all of which were journal articles. Detailed retrieval process can be referred in Figure 1.

### 3.2. Basic Characteristics and Risk of Bias Assessment of the Selected Literature

The 19 articles were published from 2015 to 2021, with a total of 1,707 cases. Among them, there were 853 cases allocated to experimental group and the remaining 854 cases assigned to control. Both groups were comparable at baseline (Table 1). After the assessment of risk of bias, the findings were presented (Figure 2). The randomization method in one study was incorrect and evaluated as high risk, and two studies did not specify their randomization methods which were evaluated as unclear. The randomization methods in the remaining studies were correct and assessed as low risk. None of the articles mentioned allocation concealment and were evaluated as unclear. Except for one study that was not explicitly blinded and evaluated as unclear, all included literature was not blinded to study participants and outcome measures, with implementation bias as high risk. Except for one study that mentioned shedding cases and was evaluated as low risk, the cause of shedding was not reported, and the loss of follow-up bias was unclear. The outcomes listed were consistent with the outcome reports, and thus, the reporting bias was low risk. Other bias was unclear.

### 3.3. Meta-Analysis Results

#### 3.3.1. Mayo Score

Four studies involving 298 people were included, with the heterogeneity of *I*^2^ = 78% (*P* = 0.004), so we adopted the random-effects model. The Mayo score in the experimental group was markedly decreased versus control (MD = −1.94, 95% CI (-2.69, -1.19), *P* < 0.00001), and the difference between both groups was regarded statistically significant, as shown in Figure 3. These results indicated that the Mayo score of Bifidobacterium quadruple viable bacteria combined with mesalamine against UC was decreased as compared to control; thus, the degree of disease activity after combined treatment was lower than that of control.

#### 3.3.2. Total Efficiency

A total of 16 studies were included, including 1,513 people. Heterogeneity test showed *I*^2^ = 0% (*P* = 1.00), so we employed the fixed-effects model. The incidence of the total effective number of individuals was increased in the experimental group versus control (OR = 5.10, 95% CI (3.53, 7.38), *P* < 0.00001), indicating the presence of statistical difference of both groups, as shown in Figure 4(a). According to Egger's test (*P* = 0.001) and Begger's test (*P* = 0.001), certain publication bias existed, as shown in Figure 4(b). The combined effect size RR and confidence interval were calculated by fitting and supplementing the fixed-effects model of six articles, and the conclusions before and after the trim and filling method were consistent (Figure 4(c)).

#### 3.3.3. Interleukins

A total of 15 studies were included with 1,436 participants studied. We adopted a random-effects model as the heterogeneity results showed *I*^2^ = 97% (*P* < 0.00001). Interleukin level in the experimental group decreased markedly versus control (SMD = −0.87, 95% CI (-1.59, -0.15), *P* < 0.00001). The results were considered statistically significant difference between both groups, suggesting that Bifidobacterium quadruple viable bacteria combined with mesalamine had a mitigating effect on the release of inflammatory factors in UC (Figure 5(a)). Next, we carried out a subgroup analysis, among which 10 studies were included in the interleukin-8 group with 957 participants. A random-effects model was adopted as *I*^2^ = 93% (*P* <0.00001) for heterogeneity. The level of interleukin-8 in the experimental group declined substantially vs. control (SMD = −1.79, 95% CI (-2.36, -1.12), *P* < 0.00001), implying that there was a statistically significant difference. Five studies were included and 479 subjects were studied in the interleukin-4 group, and a random-effects model was utilized since *I*^2^ = 77% (*P* < 0.001) for heterogeneity. The level of interleukin-4 was also greatly increased in the experimental group vs. control (SMD = 1.00, 95% CI (0.60, 1.41), *P* < 0.00001). The difference was regarded statistically significant. According to Egger's test (*P* = 0.038) and Begger's test (*P* = 0.020), publication bias presented (Figure 5(b)); thus, the trim and filling method was further applied. The combined effect size RR and confidence interval calculated by the random-effects model reached the same conclusion before and after the trim and filling, with no literature to supplement, as shown in Figure 5(c).

#### 3.3.4. TNF-*α*

Seven studies involving 688 participants were included. A random-effects model was utilized as heterogeneity indicating *I*^2^ = 96% (*P* < 0.00001), and the experimental group had a decreased TNF-*α* level as compared to control (MD = −7.11, 95% CI (-9.23, -5.00), *P* < 0.00001), and both groups presented statistical difference **(**see Figure 6(a)). However, Egger's test (*P* = 0.764) and Begger's test (*P* = 0.753) revealed no significant publication bias, as shown in Figure 6(b).

#### 3.3.5. Hypersensitive C-Reactive Protein (hs-CRP)

A total of ten studies were included, with 953 people studied. After the determination of heterogeneity, a random-effects model was adopted as *I*^2^ = 95% (*P* < 0.00001). The test results revealed a marked increase in the levels of hs-CRP in the experimental group as compared to control (MD = −3.26, 95% CI (-4.28, -2.25), *P* < 0.00001), and the presence of statistical difference was considered, as shown in Figure 7(a). According to Egger's test (*P* = 0.283) and Begger's test (*P* = 0.092), publication bias was not significant, as shown in Figure 7(b).

#### 3.3.6. ox-LDL

Three studies including 268 patients were included, with the heterogeneity of *I*^2^ = 0% (*P* =0.59), and the fixed-effects model was employed. The test findings revealed a marked decrease in the levels of ox-LDL in the experimental group vs. control (MD = −14.46, 95% CI (-17.20, -11.72), *P* < 0.00001), and the two groups presented statistical difference, as shown in Figure 8.

#### 3.3.7. LPO

A total of six studies were included, with 588 people studied. After heterogeneity determination, we employed the random-effects model as *I*^2^ = 96% (*P* < 0.00001). Our findings revealed a substantial decreased in the level of LPO in the experimental group vs. control (MD = −3.55, 95% CI (-4.70, -2.39), *P* < 0.0001), as well as the presence of statistical difference, as shown in Figure 9.

#### 3.3.8. SOD

Five studies with 496 patients were included for heterogeneity test. We then adopted the random-effects model as *I*^2^ = 90% (*P* <0.00001). The experimental group revealed a marked increase in the level of SOD vs. control (SMD = 1.68, 95% CI (1.02, 2.35), *P* < 0.00001), which was assumed the presence of statistical difference, as shown in Figure 10.

#### 3.3.9. Adverse Reactions

A total of fourteen studies were included, involving 1,221 patients. With the heterogeneity of *I*^2^ = 33% (*P* = 0.11), a fixed-effects model was adopted. Adverse reactions in the experimental group were substantially less than control (OR = 0.43, 95% CI (0.28, 0.66), *P* = 0.001), implying that the two groups presented statistical difference, see Figure 11(a). Egger's test (*P* = 0.744) and Begger's test (*P* = 0.827) demonstrated no significant publication bias, as shown in Figure 11(b).

## 4. Discussion

UC is a refractory disease, the incidence of which is on the rise worldwide [32], and there is a lack of specific and effective treatments at present. Currently, drugs in the 5-ASA class are preferred for mild to moderate UC, whereas efficacy varies from person to person. With progressive medical advances, UC and intestinal flora imbalance have been found to be associated [33]. Most studies have shown that probiotics by modulating the intestinal tract are effective in the treatment of UC [34, 35]. Intestinal flora also exerts vital roles for UC development and progression. Current studies have found that the imbalance of the ratio of beneficial and harmful bacteria in the intestinal tract may promote UC incidence [36], prolong the remission time of clinical symptoms of this disease, and reduce the duration of remission after treatment. It has been shown that Bifidobacterium quadruple viable bacterium significantly improves the levels of inflammatory factors and lipid peroxidation status in UC [37]. Multiple randomized controlled trials of Bifidobacterium quadruple viable bacteria in combination with mesalamine in UC treatment have confirmed much benefits from Bifidobacterium quadruple viable bacteria combined with mesalamine in treating UC [29, 30, 38–41].

This meta-analysis showed that mesalamine combined with Bifidobacterium quadruple viable bacteria was significantly superior to mesalamine alone in improving the Mayo score, reducing proinflammatory factor release, and improving lipid peroxidation damage in managing UC from mild to moderate stages, which could also effectively improve the clinical efficacy. In terms of safety, adverse reactions were apparently less by introducing combined medication in the disease control than control. Moreover, this combined therapy was more reliable than the single agents. However, whether the combination of drugs can achieve long-term therapeutic effects still needs further verification.

The strengths of this meta-analysis are as follows: (1) all included studies were RCTs; (2) multiple observational indicators including efficacy and safety were included; (3) currently, there is an increasing trend of prevalence in Asia, and this study has included Chinese literature to study the Asian population and found that both effectiveness and safety of Bifidobacterium quadruple viable bacteria combined with mesalamine were better than that of the group with the single agent in Chinese patients with UC. Nevertheless, this meta-analysis still has some limitations. Most studies did not mention double-blind methods. Although six databases in English and Chinese were systematically searched, large sample and multicenter experiments were still lacking. The current work provided a clinical reference for the application of Bifidobacterium quadruple viable bacteria combined with mesalamine against UC treatment.

## 5. Conclusion

In conclusion, the current meta-analysis shows that Bifidobacterium quadruple viable bacteria combined with mesalamine has a satisfactory effect in the treatment of UC in China, and its safety is better than that of mesalamine or Bifidobacterium quadruple viable bacteria alone. However, randomized controlled trials with standardized designs and large sample sizes are still needed for further validation.

## Figures and Tables

**Figure 1:** Flow chart of literature search.

**Figure 2:** Bibliographic risk assessment chart.

**Figure 3:** Forest plot of the Mayo score.

**Figure 4:** Forest plot of total efficiency (a). Begger's funnel plot of publication bias for total efficiency (b). Filled funnel plot of total efficiency (c).

**Figure 5:** Forest plot of interleukins (a). Begger's funnel plot of publication bias for interleukins (b). Filled funnel plot of interleukins (c).

**Figure 6:** Forest plot of TNF-*α* (a). Begger's funnel plot of publication bias for TNF-*α* (b).

**Figure 7:** Forest plot of hs-CRP (a). Begger's funnel plot of publication bias for hs-CRP (b).

**Figure 8:** Forest plot of ox-LDL.

**Figure 9:** Forest plot of LPO.

**Figure 10:** Forest plot of SOD.

**Figure 11:** Forest plot of adverse reactions (a). Begger's funnel plot of publication bias for adverse reactions (b).

**Table 1:** List of basic features of literature.

	Age (years old)		Number of samples		Interventions		Duration of treatment (month)	Outcomes
	E	C	E	C	E	C		
Zhang J [37]	36 ± 6.9	36 ± 8.9	38	38	M+QB	M	2	1; 2; 3; 4; 5
Zhang Y [37]	44.6 ± 5.8	45.3 ± 5.5	55	55	M+QB	M	2	2; 4; 5; 6; 7; 8; 9; 10
Che J [42]	38.4 ± 5.7	38.6 ± 5.9	37	37	M+QB	M	12	2; 4; 5; 6; 10
Cheng P [43]	36.12 ± 6.52	35.42 ± 6.25	30	30	M+QB	M	1	2; 4; 5; 10
Guo ET [44]	25.74 ± 2.15	25.93 ± 2.27	65	65	M+QB	M	1.5	4; 6; 8; 9; 10
Hou J [45]	44.26 ± 3.74	43.68 ± 3.41	43	43	M+QB	M	2	1; 2; 3; 4; 5; 6
Hou LL [25]	41.65 ± 8.12	41.84 ± 8.03	79	79	M+QB	M	2	2; 5; 6; 10
Jin Y [46]	34.35 ± 4.12	34.06 ± 4.08	52	52	M+QB	M	2	4; 6; 10
Pang YM [47]	26.14 ± 3.05	27.25 ± 4.62	51	51	M+QB	M	1.5	6; 8; 9
Ruan RH [48]	41.6 ± 6.6	41.3 ± 7.3	42	42	M+QB	M	1.5	2; 3; 4; 5; 6
Sun ZY [49]	50.19 ± 2.22	50.16 ± 2.24	44	44	M+QB	M	2	5; 6; 8; 9
Tan WK [50]	38.96 ± 9.02	39.05 ± 8.89	25	25	M+QB	M	3	2; 5; 6
Wang SJ [51]	57.1 ± 9.5	58.3 ± 7.6	26	26	M+QB	M	1	5; 10
Wang YG [52]	45.00 ± 4.50	45.50 ± 4.00	75	75	M+QB	QB	1.5	2; 3; 4; 5; 6
Wang YD [53]	40.7 ± 4.8	41.2 ± 5.1	41	42	M+QB	M	1.5	2; 3; 4; 5; 6
Wang YB [54]	38.98 ± 4.23	40.12 ± 4.05	46	46	M+QB	M	2	6; 7; 8
Xu JY [55]	41.9 ± 4.6	42.6 ± 5.0	36	36	M+QB	M	1.5	5; 6; 7; 8; 9
Yue YY [56]	35.8 ± 6.6	35.5 ± 6.8	32	32	M+QB	M	1	1; 5; 6
Zheng Y [57]	35.22 ± 6.06	36.08 ± 5.43	36	36	M+QB	M	2	1; 2; 6

Note: E: test group; RCT: randomized controlled trial; C: control group; M: mesalamine; QB: Bifidobacterium quadruple viable bacteria; 1: Mayo Score; 2: hs-CRP hypersensitive C-reactive protein; 3: IL-4: Interleukin-4; 4: IL-8: Interleukin-8; 5: adverse reactions; 6: total efficiency; 7: ox-LDL: oxidized low density lipoprotein; 8: LPO: lipid peroxide; 9: SOD: superoxide dismutase; 10: TNF*α*: tumor necrosis factor.

## Data Availability

All data generated or analyzed are available from the corresponding author on reasonable request.
